The article "Expression of microRNA-497 and its prognostic significance in human breast cancer" was retracted in 2015. Reasons: misconduct by a third party; compromised peer review.

# Expression of microRNA-497 and its prognostic significance in human breast cancer

**DOI:** 10.1186/1746-1596-8-172

**Published:** 2013-10-21

**Authors:** Shaohua Wang, Hanjun Li, Jingjie Wang, Dan Wang

**Affiliations:** 1 Department of General Surgery, Jinling Hospital, School of Medicine, Nanjing University, 315 Zhongshan East Road, Nanjing, Jiangsu 210002, PR China

**Keywords:** MicroRNA-497, Breast cancer, qRT-PCR, Disease-free survival, Overall survival

## Abstract

**Objective:**

Dysregulation of microRNAs (miRNAs) plays critical roles in tumor progression. The aim of this study was to investigate the clinicopathologic and prognostic significance of miR-497 expression in human breast cancer (BC).

**Methods:**

Taqman qRT-PCR assay was performed to detect the expression of microRNA (miR)-497 in 30 pairs of BC tissues and corresponding noncancerous breast tissues. Additionally, the expression of this miRNA was detected in another 128 BC tissues and its correlations with clinicopathologic features of patients were analyzed. Kaplan-Meier analyses were used to assess survival of patients. Univariate and multivariate analyses were performed using the Cox proportional hazards model to analyze the prognostic significance of miR-497 expression.

**Results:**

Our data indicated that the relative level of miR-497 expression in BC tissues was significantly lower than that in corresponding noncancerous breast tissues (*P* = 0.0046). Of 128 BC patients, 74 (57.8%) were placed in the high-miR-497 group and 54 (42.2%) were placed in the low-miR-497 group. By statistical analyses, low miR-497 expression was observed to be closely correlated with higher differentiation grade, positive HER-2 expression, higher incidence of lymph node metastasis and advanced clinical stage. Moreover, patients with high miR-497 expression had better 5-year disease-free and overall survival compared with the low miR-497 group (*P* = 0.0124 and 0.0018, respectively). Univariate and multivariate analyses indicated that low miR-497 expression was an independent poor prognostic factor for BC patients.

**Conclusions:**

Our data provided the first evidence that downregulation of miR-497 was correlated with BC progression, and miR-497 might be a potential molecular biomarker for predicting the prognosis of patients.

**Virtual slides:**

The virtual slide(s) for this article can be found here: http://www.diagnosticpathology.diagnomx.eu/vs/2025828761093488

## Introduction

Breast cancer (BC), the top cancer in women both in the developed and the developing world, has been a leading cause of death among women in China, with 1.1 million new cases annually [1]. Although improvements in early detection and treatment have decreased breast cancer mortality rates in recent years, prevention and therapy of breast cancer remain a major public health concern [2]. China’s breast cancer mortality has doubled over the past 30 years. BC is a heterogeneous disease with respect to molecular alteration, cellular composition, and clinical outcome. Breast carcinogenesis is a multistep process characterized by genetic and epigenetic alterations that influence key cellular pathways involved in growth and development [3]. Therefore, a better understanding of the molecular mechanisms involved in BC initiation and progression will likely contribute to providing useful prognostic biomarker and therapeutic target for BC therapy.

The article "Expression of microRNA-497 and its prognostic significance in human breast cancer" was retracted in 2015. Reasons: misconduct by a third party; compromised peer review.

MiRNAs are a class of small non-coding RNAs (~22 nt) which are involved in the regulation of gene expression by inducing mRNA degradation or repressing mRNA translation [4,5]. Increasing evidence indicates that miRNAs play critical roles in many human biological and pathological processes such as growth, apoptosis, development and tumorigenesis [6-10]. These tumor-related miRNAs function as tumor suppressors or oncogenes and modulate many aspects of carcinogenesis, including cell proliferation, cell-cycle control, metastasis and angiogenesis [11-13]. Recently, the correlations of dysregulated miRNAs with human BCs are increasingly reported. By microarray and Northern blot analyses, Iorio and his colleagues reported that miRNAs were aberrantly expressed in human breast cancer and the overall miRNA expression could clearly separate normal versus cancer tissues, with the most significantly deregulated miRNAs being mir-125b, mir-145, mir-21, and mir-155 [14]. Using a bead-based flow cytometric miRNA expression profiling method, Blenkiron’ et al. identified 133 miRNAs expressed in human breast tumors, which could be used to classify breast cancer into prognostic molecular subtypes [15]. Lerebours’ et al. showed that a 5-miRNA signature comprising miR-421, miR-486, miR-503, miR-720 and miR-1303 was shown to be predictive for inflammatory BC phenotype with an overall accuracy of 89% [16]. These data clearly indicate that specific miRNA expression patterns are associated with the biological and clinical properties of human BCs. However, there have been a limited number of studies on the potential of miRNAs used for prognostic biomarkers and therapeutic molecular targets in BC. Here, the focus is on miR-497, which has been reported to be downregulated in a variety of malignant tumors, including cervical cancer, colorectal cancer, and prostate cancer [17-19]. By analysis of the genome-wide expression profiling of miRNAs, Yan and his colleagues showed that seven miRNAs of hsa-miR-497, hsa-miR-31, hsa-miR-355, hsa-miR-320, rno-mir-140, hsa-miR-127 and hsa-miR-30a-3p were significantly downregulated in BC [20]. Additionally, Shen’ et al. reported that miR-497 could induce apoptosis of breast cancer cells by targeting Bcl-w [21]. However, the prognostic significance of miR-497 in BC is not fully understood.

The article "Expression of microRNA-497 and its prognostic significance in human breast cancer" was retracted in 2015. Reasons: misconduct by a third party; compromised peer review.

In the present study, qRT-PCR assay was performed to detect the expression of miR-497 in BC and corresponding noncancerous breast tissues. Moreover, the correlations of miR-497 expression with clinicopathologic features of BC patients were statistically analyzed. Finally, we determined the potential role of miR-497 in BC prognostic prediction. Our data showed that miR-497 was significantly downregulated in BC tissues and could be served as a potential molecular biomarker for the prediction of poor prognosis.

## Methods and materials

### Patients and tissue samples

A total of 128 BC tissues, 30 paired BC and corresponding noncancerous breast tissues were collected directly from surgery after removal of the necessary amount of tissue for routine pathology examination at the Department of Pathology, Jinling or Xijing Hospital between 2003 and 2005. The tissues were immediately frozen in liquid nitrogen after surgical removal and stored at -80°C until use. None of the patients recruited in this study had undergone preoperative chemotherapy or radiotherapy. The characteristics of patients were shown in Table 1. Informed written consent was obtained from all patients. The tumors were frozen at -80°C in a guanidinium thiocyanate solution. The Chinese Medical Association Society of Medicine’s Ethics Committee approved all aspects of this study in accordance with the Helsinki Declaration.

**Table 1:** Correlations of miR-497 expression with clinicopathologic features of BC patients

	**miR-497 expression**		
**Clinicopathologic features**	**High (n = 74)**	**Low (n = 54)**	***P*-value**
Age (years)			0.204
≤50	44	38	
>50	30	16	
Tumor size (cm)			0.777
≤2.0	32	22	
>2.0	42	32	
Differentiation grade			0.005^*^
G1 + 2	46	20	
G3	28	34	
Histological type			0.078
Ductal	50	44	
Lobular	24	10	
ER status			0.590
Negative	34	21	
Positive	44	33	
PR status			0.598
Negative	18	11	
Positive	56	43	
HER-2 status			0.024^*^
Negative	49	25	
Positive	25	29	
Lymph node metastasis			0.001^*^
Absent	47	18	
Present	27	36	
Clinical stage			0.010^*^
I + II	43	19	
III	31	35	

^*^Statistically significant difference (*P* < 0.05). *ER* estrogen receptor;

*PR* progesterone receptor, *HER-2* c-erbB-2.

### Extraction of total RNA

Total RNA isolation from tissues was performed using mirVana miRNA Isolation Kit (Applied Biosystems/Ambion, Austin, TX, USA) according to the methods described previously [22]. RNA concentrations were measured using the SPECTRAmax microplate spectrophotometer (Molecular Devices Corp).

The article "Expression of microRNA-497 and its prognostic significance in human breast cancer" was retracted in 2015. Reasons: misconduct by a third party; compromised peer review.

### Taqman quantitative reverse transcription (qRT)-PCR detection of miR-497 expression

The cDNA was synthesized from 5 ng of total RNA by using the Taqman miRNA reverse transcription kit (Applied Biosystems, Foster City, CA), and the expression levels of miR-497 were quantified by using miRNA-specific TaqMan MiRNA Assay Kit (Applied Biosystems). qRT-PCR was performed by using the Applied Biosystems 7500 Sequence Detection system. The expression of miRNA was defined based on the threshold cycle (Ct), and relative expression levels were calculated as 2^-[(Ct of miR-497)-(Ct of U6)]^ after normalization with reference to expression of U6 small nuclear RNA.

### Statistical analysis

All statistical analyses were carried out using the SPSS 17.0 software package (SPSS, Chicago, IL, USA). The data were presented as the mean ± SD. The Chi-squared test was used to investigate the significance of miR-497 expression as correlated with clinicopathologic features in BC. Disease-free and overall survival curves were plotted using the Kaplan-Meier method and were evaluated for the statistical significance using a log-rank test. The significance of different variables with respect to survival was analyzed using the univariate and multivariate Cox proportional hazards model. Differences were considered statistically significant when *P* < 0.05.

## Results

### MiR-497 was remarkably downregulated in human BC tissues

Taqman qRT-PCR assay was performed to detect the expression of miR-497 in 30 pairs of BC and corresponding noncancerous breast tissues. The expression of miR-497 in 26 cases of BC tissues was downregulated in comparison with that in corresponding noncancerous breast tissues, but the expression of miR-497 was upregulated in only 4 cases of BC tissues (Figure 1A). It was shown that the mean expression level of miR-497 in BC tissues (mean ± SD: 1.23 ± 0.63) was remarkably lower than that in noncancerous breast tissues (mean ± SD: 2.89 ± 0.34; *P* = 0.0046; Figure 1B).

**Figure 1:** **Taqman qRT-PCR detection of relative miR-497 expression in tissue samples. A**. qRT-PCR was performed to respectively detect the relative miR-497 expression in 30 pairs of BC and corresponding noncancerous breast tissues. **B**. The mean expression level of miR-497 in BC tissues was significantly lower than that in corresponding noncancerous breast tissues (*P* = 0.0046). U6 snRNA was used as an internal control. Each assay was performed at least in triplicate. Corresponding *P* values analyzed by *t*-tests are indicated. T: BC tissues; N: noncancerous breast tissues.

The article "Expression of microRNA-497 and its prognostic significance in human breast cancer" was retracted in 2015. Reasons: misconduct by a third party; compromised peer review.

### Correlations of miR-497 expression with clinicopathologic features of BC patients

To further investigate the correlations of miR-497 with various clinicopathologic features of BC patients, the relative expression of miR-497 was determined in another 128 cases of BC tissue samples. The median value of miR-145 in all BC tissues was 1.46 and used as a cutoff value, and all patients were divided into two groups: high-miR-497 expression group (≥1.46; n = 74; mean ± SD: 2.04 ± 0.38) and low-miR-497 expression group (<1.46; n = 54; mean ± SD: 0.45 ± 0.28). Then, the correlations of miR-497 expression with clinicopathologic features of patients were statistically analyzed. As shown in Table 1, low miR-497 expression was observed to be closely correlated with higher differentiation grade, positive HER-2 expression, higher incidence of lymph node metastasis and advanced clinical stage (*P* = 0.005, 0.024, 0.001 and 0.010, respectively). However, there were no significant correlations between miR-497 expression and other clinicopathologic factors including age, tumor size, histological type, ER and PR status (*P* = 0.204, 0.777, 0.078, 0.590 and 0.598, respectively).

### Correlations of miR-497 expression with disease-free survival (DFS) and overall survival (OS) of BC patients

To further investigate the correlation of miR-497 expression with survival of BC patients, Kaplan-Meier analyses were performed. As shown in Figure 2A, the 5-year DFS of low-miR-497 expression group (60.4%) was significantly shorter than that of high-miR-497 expression group (81.2%; *P* = 0.0124). Moreover, the 5-year OS of low-miR-497 expression group (57.3%) was significantly shorter than that of high-miR-497 expression group (71.2%; *P* = 0.0018) (Figure 2B). These results indicated that downregulation of miR-497 might be correlated with poor survival of BC patients.

**Figure 2:** **Kaplan-Meier survival curves of BC patients. A**. The 5-year DFS of BC patients with high miR-497 expression was significantly higher than that of those patients with low miR-497 expression (*P* = 0.0124). **B**. The 5-year OS of BC patients with high miR-497 expression was significantly higher than that of those patients with low miR-497 expression (*P* = 0.0018). The *P*-value was calculated using the log-rank test between patients with high- and low-fold changes.

### Univariate and multivariate determination of prognostic factors in BC patients

Next, univariate analyses were performed to evaluate the expression of miR-497 and other clinicopathologic features on prognosis of BC patients. As shown in Table 2, it was observed that miR-497 expression, along with age, tumor size, differentiation grade, histological type, ER status, PR status, HER status, lymph node metastasis and clinical stage, was responsible for efficacy of surgical treatment in BC patient, by indicating that status of miR-497 expression was significantly correlated with DFS (*P* = 0.005) and OS (*P* = 0.036) of BC patients. Furthermore, multivariate analyses were performed to evaluate those clinicopathogic features significant in univariate analyses (tumor size, differentiation grade, lymph node metastasis, clinical stage and status of miR-497 expression). It was shown that miR-497 expression was an independent molecular biomarker for the predicting of DFS (HR: 1.535, 95% CI: 1.127-2.337, *P* = 0.016) and OS (HR: 2.123, 95% CI: 1.836-3.015, *P* = 0.008) in BC patients (Table 3).

The article "Expression of microRNA-497 and its prognostic significance in human breast cancer" was retracted in 2015. Reasons: misconduct by a third party; compromised peer review.

**Table 2:** Univariate analyses of different prognostic factors in BC patients

	**Disease-free survival**		**Overall survival**	
**Variables**	**HR (95% CI)**	***P*-value**	**HR (95% CI)**	***P*-value**
Age (years)	1.341 (0.607-1.711)	0.316	1.503 (0.733-2.012)	0.618
Tumor size (cm)	2.278 (1.566-2.791)	0.008^*^	1.808 (1.127-2.443)	0.016^*^
Differentiation grade	2.334 (1.789-2.882)	0.022^*^	2.055 (1.726-3.404)	0.001^*^
Histological type	0.802 (0.477-1.682)	0.358	1.022 (0.799-1.501)	0.207
ER status	1.563 (0.815-1.921)	0.188	0.865 (0.699-1.118)	0.295
PR status	0.855 (0.429-1.277)	0.098	1.510 (0.719-2.121)	0.411
HER-2 status	1.777 (0.892-1.954)	0.301	1.221 (0.669-1.443)	0.189
Lymph node metastasis	3.122 (1.778-3.828)	0.017^*^	2.011 (1.548-2.817)	0.038^*^
Clinical stage	1.718 (1.150-2.203)	0.008^*^	1.823 (1.199-2.458)	0.014^*^
MiR-497 expression	2.340 (1.782-2.695)	0.005^*^	1.504 (1.285-1.914)	0.036^*^

^*^P < 0*.*05. *Abbreviations*: *HR* hazard ratio, *95% CI,* 95% confidence interval, *ER* estrogen receptor, *PR* progesterone receptor, *HER-2* c-erbB-2.

**Table 3:** Mulivariate analyses of different prognostic factors in BC patients

	**Disease-free survival**		**Overall survival**	
**Variables**	**HR (95% CI)**	***P*-value**	**HR (95% CI)**	***P*-value**
Tumor size (cm)	1.660 (0.875-1.914)	0.115	0.707 (0.680-1.188)	0.073
Differentiation grade	1.146 (0.794-1.326)	0.204	1.522 (0.891-1.927)	0.163
Lymph node metastasis	2.102 (1.377-2.456)	0.009^*^	1.749 (1.087-2.514)	0.011^*^
Clinical stage	3.071 (2.318-3.549)	0.021^*^	2.362 (1.693-2.720)	0.037^*^
MiR-497 expression	1.535 (1.127-2.337)	0.016^*^	2.123 (1.836-3.015)	0.008^*^

^*^P < 0*.*05. *Abbreviations*: *HR* hazard ratio, *95% CI* 95% confidence interval.

## Discussion

As different cancer therapies are effective in different subgroups of patients, there is a tremendous need for novel predictive and prognostic markers to improve the outcomes of cancer patients [23]. BC is a group of heterogeneous diseases that show various biological and clinical characteristics. Patient management is currently based on easily identifiable clinical and pathological characteristics, which only partially reflect disease heterogeneity. Many principal factors, such as patient age, status of axillar lymph nodes, tumor size, histological traits, status of hormonal receptors and HER2, have been used for the prediction of the prognosis of BC patients for many years [24,25], but their roles in determining the individual risk level of the patient are quite limited. Therefore, it is still needed to exploit clinically useful, readily available prognostic markers in the management of BC.

The article "Expression of microRNA-497 and its prognostic significance in human breast cancer" was retracted in 2015. Reasons: misconduct by a third party; compromised peer review.

MiRNAs, important regulators of mRNA and protein expression, are emerging as important modulators of essential biological functions, including cellular development, apoptosis, metabolism and oncogenesis [26]. It is estimated that miRNAs may regulate up to a third of the human genome. They also represent a novel biological entity with potential value as tumour biomarkers, which can improve diagnosis, prognosis, and monitoring of treatment response for human cancers [27,28]. Application of the potential role of miRNAs as molecular biomarkers in human cancer is increasingly supported by the large number of studies conducted in different cancers, including BC [29,30]. Tang’ et al. reported that high miR-27a expression was associated with poor overall survival in patients with breast cancer, suggesting that miR-27a could be a valuable marker of breast cancer progression [31]. By a meta-analysis, Hong’ et al. indicated that high expression of miR-210 could predict poor survival in patients with breast cancer [32]. By screening the expression levels of 754 human miRs using miR arrays in 16 breast tumor samples from 8 cases with local recurrence and 8 cases without local recurrence, Zhou and his colleagues reported that microRNA-9 could be used as a potential biomarker for breast cancer local recurrence and tumor estrogen receptor status [33]. As the stability of miRs and their detection in circulation, the miRNAs in body fluids, such as serum and plasma, open up the possibility of using them as noninvasive biomarkers in breast cancer [34,35]. MiR-497, identified from the microRNA cluster site at chromosome 17p13.1, has been reported to function as a tumor suppressor in a variety of human cancers, including non-small cell lung cancer, hepatocelluar cancer, neroblastoma, colorectal cancer and breast cancer [18,21,36-38]. Meanwhile, it was also reported that miR-497 could modulate multidrug resistance of human cancer cell lines by targeting Bcl-2 [39]. In human cervical cancer, low miR-497 expression appeared to be an unfavorable prognostic factor for patients [17]. By analysis of the expression of 319 microRNAs in 9 primary human male breast tumors and in epithelial cells from 15 male gynecomastia specimens, Lehmann and his colleagues showed that miR-145 and miR-497 were identified as most prominently down-regulated in male BC [40]. However, the status of miR-497 expression in female BC and its prognostic roles are unclear. Thus, the aim of this study was to investigate the correlations of miR-497 expression with clinicopathologic features and prognosis of BC patients.

The article "Expression of microRNA-497 and its prognostic significance in human breast cancer" was retracted in 2015. Reasons: misconduct by a third party; compromised peer review.

Here, we first detect the expression of miR-497 in 30 pairs of BC and corresponding noncancerous breast tissues, and showed that the relative expression level of miR-497 in BC was significantly lower than that in noncancerous breast tissues. Then, we detected the expression of miR-497 in another 128 cases of BC tissues and analyzed its clinicopathologic and prognostic significance. Our results indicated that status of miR-497 expression in tissues was significantly correlated with tissue differentiation grade, HER-2 status, incidence of lymph node metastasis and clinical stage of BC patients. It was observed that patients with low miR-497 expression showed poorer differentiation grade, higher incidence of lymph node metastasis and advanced clinical stage, suggesting that downregulation of miR-497 played an important role in BC progression. Interestingly, low miR-497 expression was found to be correlated with positive HER-2 expression. In previous study, type I insulin-like growth factor receptor (IGF-1R) was identified as a functional and direct target of miR-497 in colorectal cancer and cervical cancer [17,18], and downregulation of miR-497 could lead to the overexpression of IGF-1R, which leads to malignant transformation and tumor development [41]. The IGF/IGF-1R pathway has also been shown to have extensive cross-talk with epidermal growth factor receptor (EGFR), and human epidermal growth factor receptor 2 (HER-2) signaling pathways [42]. Thus, whether downregulation of miR-497 might lead to the activation of HER-2 by inducing upregulation of IGF-1R in human BC is unclear and remains to be elucidated in future studies. Then, we analyzed the correlation of miR-497 expression with prognosis of BC patients, and found that patients with high miR-497 expression showed better DFS and OS than those with low miR-497 expression. More importantly, both the univariate and multivariate survival analyses demonstrated that low miR-497 expression was correlated with shorter OS and DFS in BC, which was also consistent with the prognostic significance of miR-497 in other human malignancies, such as cervical cancer and neuroblastoma. These results indicated that miR-497 might be an important modulator involved in BC development.

The article "Expression of microRNA-497 and its prognostic significance in human breast cancer" was retracted in 2015. Reasons: misconduct by a third party; compromised peer review.

Taken together, the current study indicates that miR-497 is downregulated in BC tissues and might be an independent molecular biomarker for predicting the prognosis of BC patients. Of course, this study has several limits. First, as the number of patients in this study is smaller, a larger case population is needed to confirm the prognostic value of miR-497 expression in BC. Second, as formalin-fixed, paraffin-embedded tissues display (FFPE) degradation of nucleic acids if compared to fresh materials, the HOPE-technique with laser microdissection represents a novel tool for future tissue-based studies described recently [43]. Finally, further investigation of the cell biology of miR-497 and its potential as a therapeutic target in BC are clearly warranted.

## Competing interests

The authors declare that they have no competing interests.

## Authors’ contributions

SHW and HJL designed the study, carried out the experiments and drafted the manuscript; HJL, JJW and DW participated in the experiments and data analysis. All authors read and approved the final manuscript.
